# B7-H4 Expression in Precancerous Lesions of the Uterine Cervix

**DOI:** 10.1155/2021/5857092

**Published:** 2021-10-05

**Authors:** Qianqian Zhang, Liju Zong, Hui Zhang, Wei Xie, Fan Yang, Wenwen Sun, Baoxia Cui, Youzhong Zhang

**Affiliations:** ^1^Department of Obstetrics and Gynecology, Qilu Hospital, Cheeloo College of Medicine, Shandong University, China; ^2^Department of Obstetrics and Gynecology, The Second Affiliated Hospital of Shandong First Medical University, China; ^3^Department of Pathology, Peking Union Medical College Hospital, Chinese Academy of Medical Sciences, China; ^4^Department of Emergency, The Second Affiliated Hospital of Shandong First Medical University, China; ^5^Department of Pathology, The Second Affiliated Hospital of Shandong First Medical University, China

## Abstract

Over 10% of patients diagnosed with cervical intraepithelial neoplasia (CIN) have no lesions detected in their cervical conization specimens. The purpose of this study was to determine the factors related to the absence of such lesions. We particularly sought to investigate whether the expression of B7-H4 in precancerous lesions and cancer of the uterine cervix plays a role in the presence or absence of residual lesions in conization specimens and whether this protein is associated with T cells (i.e., Foxp3^+^ regulatory T cells, CD4^+^, and CD8^+^) and interferon-*γ* production. Of the 807 patients with CIN treated by conization, 104 (12.9%) had no lesions in their conization specimens. Seventy-five of these patients were deemed the study group and were matched with 75 patients who did have CIN detected in their conization specimens (the control group). Immunohistochemistry and immunofluorescence staining were used to detect B7-H4, Foxp3, CD4, CD8, and interferon-*γ* in the 75 pairs of specimens obtained via biopsy; 20 samples were found to have chronic cervicitis, and another 20 had squamous cell carcinoma of the cervix. Menopause, the absence of human papillomavirus, low-grade histological findings, and a diagnosis of CIN1 and CIN2 on biopsy correlated with a low probability of lesions on conization specimens. B7-H4 expression was detected in 11.1% of CIN2, 46.6% of CIN3, and 70% of cervical cancer samples, but not in tissues representing chronic cervicitis or CIN1. B7-H4 expression was associated with the presence of lesions on conization specimens, increased regulatory T cells, decreased CD8^+^ T cells, and lower interferon-*γ* production. These data suggest that close follow-up and thorough reevaluation should be considered for patients diagnosed with CIN2 who are negative for B7-H4 expression on biopsy before proceeding with cervical conization.

## 1. Introduction

Cervical cancer develops through a multistep process that includes the development of low-grade squamous intraepithelial lesion (LSIL)/cervical intraepithelial neoplasia (CIN1) followed by high-grade squamous intraepithelial lesion (HSIL)/CIN2–3. High-risk human papillomavirus (HPV) infection contributes significantly to the pathogenesis of precancerous lesions and cancer of the cervix. Cervical excision is the standard treatment method for patients with CIN2–3 as well as for patients with CIN1 who have inadequate colposcopy and/or recurrent high-grade cytologic findings. Cold knife conization (CKC) and the loop electrosurgical excision procedure (LEEP) are commonly used cervical conization methods, which are safe and effective in clinical practice and can reduce the risk of cervical cancer by 95% [1, 2]. However, several observational studies have highlighted the potential adverse effects of conization on fertility and pregnancy outcomes (such as preterm delivery, premature membrane rupture, low birth weight, caesarean section, and perinatal death) when the lesions are located in the columnar epithelium, or the excised cone has to be deep, up to the internal os of the cervix [3, 4]. Notably, however, 13.8–16.5% patients with histologically confirmed CIN2–3 on a previous biopsy have no residual CIN in their final excision specimens. Therefore, it is necessary to identify factors that can predict the absence of CIN in conization specimens to avoid unnecessary treatment and unexpected complications [5].

HPV infection is self-limiting and can be eradicated by the immune response in the normal cervical microenvironment. The reduction in immune surveillance and clearance rates is an important contributor to cervical pathogenesis and development [6, 7]. To that end, B7 family members and their receptors are crucial for the regulation of antigen-specific immune responses [8]. B7 homolog 4 (B7-H4, B7x, or B7S1) is an immunoregulatory member of the B7 family that was identified recently [9–11]; this protein has been found in several tumor types, including ovarian, breast, kidney, liver, lung, spleen, thymus, and placental cancers [12]. Previous studies showed that the expression of B7-H4 in cervical cancer is associated with immunosuppression in the tumor microenvironment as well as tumor progression and poor prognosis [13, 14]. Furthermore, B7-H4 has been implicated in the inhibition of T cell-mediated immunity and downregulation of T cell response via the inhibition of T cell proliferation, cytokine production, and cell cycle progression [11, 15, 16]; these events suppress the antitumor immune function. Moreover, our previous study found that the level of serum B7-H4 was higher in patients with CIN than in healthy volunteers [14]. However, B7-H4 expression in CIN and its potential association with the presence or absence of excised conization specimens remain unknown, as does its relationship with tumor-infiltrating T lymphocytes.

The purpose of this study was to identify predictors of CIN lesion absence in cervical conization samples from patients diagnosed with CIN via biopsy, to investigate the expression of B7-H4 in CIN and cervical cancer, and to determine the association between this protein and the pathological features and T cells of the immune microenvironment.

## 2. Materials and Methods

### 2.1. Patients

A total of 807 patients who underwent either a CKC or LEEP procedure after cervical biopsy between July 2005 and December 2013 at Qilu Hospital of Shandong University (Ji'nan, China) were identified. Data were extracted from the colposcopy computer database and the hospital's patient database, which included the patients' age, menopausal status, cone lesion depth, punch biopsy histological grade, histological grade and margin status of the excised sample, and glandular involvement. This study was approved by the Institutional Review Board (KYLL-2017-560); informed consent was not required owing to its retrospective nature.

### 2.2. Tissue Samples

To evaluate whether B7-H4 expression was associated with the absence of lesions in conization specimens, we compared B7-H4 expression in lesion-absent and lesion-present groups. Seventy-five biopsy specimens from the group with absent lesions in their excised cervical samples were available for immunohistochemistry (IHC). Hence, 75 propensity score-matched patients were selected from the 703 who had lesions in their conization specimens. There were no significant differences between the matched groups in terms of age, menopause, thin-prep cytology test (TCT), punch biopsy, HPV status, margin involvement, glandular involvement, colposcopy, and excision methods. Hematoxylin-eosin-stained slides and paraffin-embedded tissues from the 75 pairs of biopsy specimens were obtained from the Department of Pathology, Qilu Hospital of Shandong University. The initial histopathological diagnoses were rereviewed by two gynecological pathologists. Additionally, 20 biopsy samples, each representing chronic cervicitis and squamous cell carcinoma (SCC) of the cervix, were used for IHC and immunofluorescence staining.

### 2.3. IHC

IHC was performed using our laboratory protocol as described previously [17–19]. Briefly, 4 *μ*m TMA serial sections were deparaffinized and subjected to heat-induced epitope retrieval with 10 mM sodium citrate (pH 6.0) at 95°C for 20 min. The endogenous peroxidase activity was quenched using a 0.3% hydrogen peroxide solution. Sections were incubated with primary antibody against B7-H4 (dilution 1 : 200, clone D1M8I, Cell Signaling Technology, Danvers, USA). Human placental tissues treated with primary antibodies were used as positive controls, while the same tissues with isotype-matched antibodies comprised negative controls.

### 2.4. Immunofluorescence

Immunofluorescence-based staining was performed to detect CD4^+^ T cells as well as CD8^+^ T cells, CD4^+^Foxp3^+^ regulatory T cells (Tregs), and interferon- (IFN-) *γ*^+^CD8^+^ T cells in cervical tissues. The slides were prepared using the same procedure as that for IHC. After blocking with 5% goat serum, slides were incubated with the following primary antibodies overnight at 4°C: rabbit anti-human Foxp3 (dilution 1 : 300, NB100-39002SS, Novus Biologicals, Littleton, CO, USA), mouse anti-human CD4 (dilution 1 : 200, NBP2-27216, Novus Biologicals), mouse anti-human CD8 alpha (dilution 1 : 200, NBP2-32836, Novus Biologicals), and rabbit anti-human IFN-*γ* (dilution 1 : 100, 8455P, Cell Signaling Technology). The secondary antibodies were goat anti-mouse IgG-phycoerythrin (dilution 1 : 1000, ab97024; ab150079) and goat anti-rabbit IgG-allophycocyanin conjugate (Abcam, Cambridge, MA, USA). After antibody removal and washing, the appropriate secondary antibody was applied, and the slides were incubated for 2 h at room temperature in the dark. Coverslips were applied to the slides using Prolong® Gold antifade reagent.

### 2.5. Image Analysis

IHC analysis was performed by two independent investigators. Brown or yellow B7-H4 staining of the membrane or cytoplasm was considered positive. Images of the various stained tissue sections were digitally photographed using a color camera (BX53; Olympus, Japan) attached to a light microscope. For B7-H4-positive samples, ×100 magnified images were captured, and the numbers of positive cells and their staining intensities were then analyzed using the Image-Pro Plus software, version 6.0 (Media Cybernetics, Silver Spring, MD, USA). For immunofluorescence staining analyses, six photographs were obtained using high-power fields (×200 magnification) per section via confocal microscopy (E2V Andor Revolution, England). The numbers of each type of T lymphocytes were autocounted using the statistical software package.

### 2.6. Statistical Analysis

Statistical analysis was performed using the SPSS version 22.0 for Windows (IBM Corp., Armonk, NY, USA). Discrete variables are expressed as the medians (ranges) and categorical variables as numbers (percentages). Analysis of categorical data was performed using the chi-square test or Fisher's exact test. Multivariate logistic regression models were used to identify variables that were independent prognostic factors; the hazard ratios were calculated as indicators of risk. Quantitative data are expressed as mean percentages ± standard deviations, and their significance was determined using Student's *t*-test or Wilcoxon rank sum test. All *P* values were two-tailed, and *P* ≤ 0.05 was considered statistically significant.

## 3. Results

### 3.1. Patient Characteristics

A total of 807 patients underwent cervical conization after first having undergone punch biopsies; their ages ranged from 21 to 62 years with a mean of 38.8 ± 8.0 years. The patients' detailed characteristics are shown in Table 1.

### 3.2. Factors Associated with the Absence of Lesions on Excised Conization Tissues

Factors associated with the absence of lesions on excised specimens are shown in Table 1. Of the 807 conization samples, 104 (12.9%) lacked lesions. Menopause, absence of HPV DNA, inadequate colposcopy sample collection, absence of glandular involvement in biopsy samples, and a conization depth ≤ 18 mm were significantly associated with the absence of lesions in excised specimens. Patients diagnosed with CIN1 and CIN2 on cervical punch biopsy, those with “negative for intraepithelial lesion or malignancy” status, those with atypical squamous cells/LSIL on TCT, and those who underwent LEEP were less likely to have lesions on their excision specimens. Neither the patients' age nor the number of biopsies during the initial colposcopy or interval between biopsy and excision was associated with the absence of lesions on excised conization tissues. Multivariate logistic regression analysis revealed that menopause and CIN2 on biopsy were independent predictors of a lack of lesions in excised conization specimens (Table 2).

### 3.3. Expression of B7-H4 in Precancerous Lesions and SCC of the Uterine Cervix

B7-H4 was detected in cervical cancer cells and in CIN2–3 epithelial cells (exhibiting a cytoplasmic/membranous staining pattern), but not in CIN1 or chronic cervicitis (Figure 1). B7-H4 expression was observed in 11.1% of the patients with CIN2, 46.7% of those with CIN3, and 70% of those with cervical cancers (Table 3). No differences in the intensity and positivity proportion of B7-H4 were observed between B7-H4-positive CIN2–3 samples and tumor samples.

B7-H4 was detected in 17.3% (13/75) of the biopsy samples from patients with absent lesions in excised conization samples and in 38.7% (29/75) of the biopsy samples from those with such lesions present; the difference was statistically significant (*P* = 0.004).

### 3.4. Correlation between B7-H4 Expression and Tumor-Infiltrating T Lymphocytes

The tumor-infiltrating T lymphocytes were mainly distributed in the surrounding matrix of cervical SCC nests and were occasionally detected in some tumoral and CIN nests.

The numbers of tumor-infiltrating CD8^+^ T cells, INF-*γ*^+^, and INF-*γ*^+^CD8^+^ T cells in B7-H4-negative samples were significantly higher than those in B7-H4-positive counterparts. However, the number of Tregs (CD4^+^Foxp3^+^) in B7-H4-positive samples was significantly higher than that in B7-H4-negative counterparts (Table 4). The numbers of CD4^+^ T cells were not significantly different between the B7-H4-negative and B7-H4-positive groups. These data indicate that B7-H4 is associated with inhibitory signals in the tumor microenvironment. Representative images of double immunofluorescence staining for CD4^+^Foxp3^+^ and IFN-*γ*^+^CD8^+^ T cells are shown in Figure 2.

## 4. Discussion

In this study, 12.9% of our patients who were diagnosed with CIN via punch biopsy (104/807) ultimately lacked lesions on their excised conization specimens. This was consistent with a rate of 16% in a previous study [20]. We also found that menopause, absence of HPV DNA, a conization depth ≤ 18 mm, low-grade findings on TCT, and CIN1 and CIN2 on biopsy correlated with the absence of lesions in the excised tissues. One explanation for the absence of CIN in conization specimens following a biopsy that diagnoses CIN is the total removal of the dysplastic lesions during the biopsy [21]. Another is that lesions embedded deep in the endocervical canal are usually not visible and may therefore be missed during cervical conization. Moreover, cervical conization may not remove the affected area in patients with small and/or peripheral transformation zones. Another possibility is the destruction of the dysplastic region by postbiopsy inflammation, spontaneous regression of the lesion, or immune system-mediated elimination after the biopsy. A previous study found that approximately 20% of CIN2–3 lesions regressed spontaneously after a confirmatory biopsy [22]. In our present study, 20.5% of the patients with CIN2 and 8.3% of those with CIN3 did not exhibit any lesions in their cervical excision specimens. The high percentage of absent lesions after a confirmed CIN2 diagnosis by biopsy suggests that women diagnosed with CIN2 may only require close follow-up and reevaluation.

B7-H4 protein is not detected in most healthy tissues but is widely expressed in various cancers. In some types of malignancies, it is associated with adverse clinical features and unfavorable prognoses [23]. Chen et al. investigated B7-H4 protein in precancerous lesions of the esophagus and found it highly expressed in 9.1% of normal tissues, 40.7% of low-grade intraepithelial neoplasia, and 81.0% of high-grade intraepithelial neoplasia. Similarly, B7-H4 was detected in HSIL and SCC in our study but not in LSIL or tissues from chronic cervicitis. These findings indicate that B7-H4 expression increases during the process of uterine cervix carcinogenesis. Furthermore, we found that negative B7-H4 expression correlates with the absence of CIN in cervical conization specimens postbiopsy. This suggests that patients with negative B7-H4 on biopsy are less likely to have lesions detected in conization specimens; therefore, unnecessary treatments such as cervical conization can be avoided and be replaced with close follow-up and thorough subsequent reevaluation.

B7-H4 expression and its association with CD8^+^ T cells, CD4^+^Foxp3^+^ Tregs, and IFN-*γ* production have been investigated in many tumors [8, 16, 24, 25]. B7-H4 expression was inversely correlated with CD8^+^ T cell infiltration in breast tumor cells and was associated with reduced activation, expansion, and cytotoxicity of CD8^+^ T cells [24, 25]. In a study of 67 patients with cervical cancer, Wang et al. found that the number of infiltrating CD8^+^ T cells in B7-H4-negative tumors was significantly higher than that in B7-H4-positive counterparts, as was their IFN-*γ* production [8]. Consistent with previous studies, we found that CD8^+^ T cells and INF-*γ*^+^CD8^+^ T cells were lower in B7-H4-positive precancerous cervical lesions. Moreover, the number of CD4^+^Foxp3^+^ Tregs was higher in our B7-H4-positive specimens than that in our B7-H4-negative ones, which reflects a previously reported positive association between Tregs and B7-H4 in ovarian cancers [16, 26]. It is worth noting that Tregs are able to trigger macrophages to secrete interleukin-6 (IL-6) and IL-10, which in turn stimulate expression of B7-H4 [26]. In our present study, IFN-*γ* secretion was decreased in B7-H4-positive samples; previous studies have shown that blocking B7-H4 enhanced the secretion of IFN-*γ* from CD4^+^ and CD8^+^ T cells [25, 27]. Podojil et al. demonstrated that the B7-H4 antibody inhibits T cell function via interleukin-10/Treg-dependent mechanisms [28]. Rahbar et al. demonstrated that IFN-*γ* upregulated B7-H4 expression on mouse embryo fibroblasts and that the upregulation of B7-H4 in tumors was T cell-dependent [29]. INF-*γ* participates in antitumor immunity by promoting the activation of macrophages and natural killer cells while enhancing the destructive potential of CD8^+^ T cells. Taken together, these data show that B7-H4 positivity is associated with a decrease in CD8^+^ T cell function and with a more immunosuppressive microenvironment in precancerous lesions and SCCs of the uterine cervix. As such, inhibiting B7-H4 using therapeutic antibodies or increasing IFN-*γ* may be potential treatment for HSIL of the cervix.

We acknowledge some limitations in our study. First, it was a retrospective investigation that produced inherent, unavoidable biases. Second, B7-H4 was detected in a relatively small size of samples. Lastly, our study was limited by its single-center nature and a lack of an independent validation cohort. Further studies from independent cohorts are needed to validate our findings.

In conclusion, we found that at least one-tenth of the patients did not have lesions in their cervical conization specimens after having undergone a diagnostic biopsy, especially those who were postmenopausal, exhibited an absence of HPV DNA, had low-grade findings on TCT, and/or were diagnosed with CIN1 and CIN2 on biopsy. Moreover, the immune checkpoint B7-H4 was detected in HSILs and SCCs but not in LSILs or cervicitis, and its expression was associated with the presence of lesions in conization specimens, increased Tregs, fewer CD8^+^ T cells, and decreased IFN-*γ* production. These data suggest that close follow-up and thorough reevaluation can be considered for patients diagnosed with CIN2 who have negative B7-H4 expression on biopsy in lieu of cervical conization.

## Figures and Tables

**Figure 1:** Expression of B7-H4 in cervical tissues. (a) Negative B7-H4 staining in chronic cervicitis, (b) positive B7-H4 staining in cervical intraepithelial neoplasia-3, and (c) positive B7-H4 staining in squamous cell carcinoma of the cervix. Magnification: ×200.

**Figure 2:** Double immunofluorescence-based staining of (a) CD4^+^Foxp3^+^ and (b) interferon (IFN)-*γ*^+^CD8^+^ T cells. Magnification: ×200.

**Table 1:** Patient characteristics as well as factors associated with the absence of lesions in excised conization tissues in patients who had undergone uterine cervical biopsies (*N* = 807).

Characteristics	Group	*N*	Lesion in excision specimens, *N* (%)		*P* value
			Present	Absent	
Age (years)	≤35	277	245 (88.4)	32 (11.6)	0.413
	>35	530	458 (86.4)	72 (13.6)	

Menopause	Yes	65	45 (69.2)	20 (30.8)	<0.001
	No	742	658 (88.7)	84 (11.3)	

Referral cytology	NILM	43	36 (83.7)	7 (16.3)	0.038
	ASCUS/LSIL	377	323 (85.7)	54 (14.3)	
	ASC-H/HSIL	210	196 (93.3)	14 (6.6)	
	Cancer	7	6 (85.7)	1 (14.3)	

Referral HPV DNA (*N* = 631)	Positive	577	501 (86.8)	76 (13.2)	0.01
	Negative	54	40 (74.0)	14 (26.0)	

Punch biopsy	CIN1	43	34 (79.0)	9 (20.9)	<0.01
	CIN2	259	206 (79.5)	53 (20.5)	
	CIN3	504	462 (91.7)	42 (8.3)	

Number of biopsies	<4	134	119 (88.8)	15 (11.2)	0.760
	4	612	532 (86.9)	80 (13.1)	
	>4	61	52 (85.2)	9 (14.8)	

Colposcopy examination (*N* = 411)	Adequacy	327	292 (89.3)	35 (10.7)	0.039
	Inadequacy	84	68 (81.0)	16 (19.0)	

Glandular involvement (*N* = 797)	Free	418	348 (83.3)	70 (16.7)	<0.01
	Involved	379	347 (91.6)	32 (8.4)	

Depth of conization	≤18 mm	333	279 (83.8)	54 (16.2)	0.022
	>18 mm	468	418 (89.3)	50 (10.7)	

Interval between biopsy and excision (months)	<1	428	370 (86.4)	58 (13.6)	0.918
	1–2	153	134 (87.6)	19 (12.4)	
	2–3	29	24 (82.8)	5 (17.2)	
	>3	30	26 (86.7)	4 (13.3)	

Conization methods	CKC	563	502 (89.2)	61 (10.8)	0.008
	LEEP	243	200 (82.3)	43 (17.7)	

CKC: cold knife conization; LEEP: loop electrosurgical excision procedure; CIN: cervical intraepithelial neoplasia; HPV: human papilloma virus; TCT: thin-prep test; ASCUS: atypical squamous cells; LSIL: low-grade squamous intraepithelial lesion; ASC-H: atypical squamous cells (cannot exclude high-grade squamous intraepithelial lesions); HSIL: high-grade squamous intraepithelial lesion; NILM: negative for intraepithelial lesion or malignancy.

**Table 2:** Multivariate logistic regression analysis of factors predictive of the absence of lesions in excised conization specimens among patients who had undergone punch biopsies.

Parameters	Hazard ratios (95% confidence interval)	*P* value
Menopause		
Yes *vs.* no	0.244 (0.107–0.554)	0.001
Punch biopsy		
CIN1 *vs.* CIN3	1.724 (0.576–5.165)	0.330
CIN2 *vs.* CIN3	2.508 (1.329–4.732)	0.005

CIN: cervical intraepithelial neoplasia.

**Table 3:** B7-H4 expression in precancerous lesions and in cancers of the uterine cervix.

Cervical tissues	*N*	B7-H4, *N* (%)	
		Positive	Negative
Cervicitis	20	0 (0.0)	20 (100)
CIN1	12	0 (0.0)	12 (100)
CIN2	63	7 (11.1)	56 (89.9)
CIN3	75	35 (46.7)	40 (53.3)
SCC	20	14 (70.0)	6 (30.0)

CIN: cervical intraepithelial neoplasia; SCC: squamous cell carcinoma. *P*-value <0.001.

**Table 4:** Correlation between B7-H4 expression and the number of infiltrating T lymphocytes and cytokines in patients with cervical disease.

T lymphocytes/cytokine	*X* ± *S*	B7-H4		*P* value
		Positive	Negative	
CD4^+^ T cells	9.67 ± 6.22	10.00 ± 8.89	9.33 ± 4.16	0.912
Tregs	11.00 ± 7.04	17.33 ± 1.53	4.66 ± 1.15	<0.001
CD8^+^ T cells	9.50 ± 9.07	2.67 ± 3.06	16.33 ± 7.51	0.043
INF-*γ*	7.83 ± 5.98	3.33 ± 4.93	12.33 ± 2.08	0.040
INF-*γ*^+^CD8^+^ T cells	6.00 ± 6.48	0.50 ± 0.70	11.50 ± 2.12	0.020

*X* ± *S*: mean ± standard deviation; INF: interferon.

## Data Availability

The relevant data used to support the findings of this study are included within the article.
